# Multi-Class Skin Problem Classification Using Deep Generative Adversarial Network (DGAN)

**DOI:** 10.1155/2022/1797471

**Published:** 2022-03-23

**Authors:** Maleika Heenaye-Mamode Khan, Nuzhah Gooda Sahib-Kaudeer, Motean Dayalen, Faadil Mahomedaly, Ganesh R. Sinha, Kapil Kumar Nagwanshi, Amelia Taylor

**Affiliations:** ^1^Department of Software and Information Systems, University of Mauritius, Reduit, Mauritius; ^2^Accenture Technology, Ebene Cyber, Mauritius; ^3^Department of Electronics and Communication Engineering, Myanmar Institute of Information Technology, Mandalay, Myanmar; ^4^Department of Computer Science and Engineering, Amity University Rajasthan, Jaipur, Rajasthan 302006, India; ^5^Malawi University of Business and Applied Sciences, Blantyre, Malawi

## Abstract

The lack of annotated datasets makes the automatic detection of skin problems very difficult, which is also the case for most other medical applications. The outstanding results achieved by deep learning techniques in developing such applications have improved the diagnostic accuracy. Nevertheless, the performance of these models is heavily dependent on the volume of labelled data used for training, which is unfortunately not available. To address this problem, traditional data augmentation is usually adopted. Recently, the emergence of a generative adversarial network (GAN) seems a more plausible solution, where synthetic images are generated. In this work, we have developed a deep generative adversarial network (DGAN) multi-class classifier, which can generate skin problem images by learning the true data distribution from the available images. Unlike the usual two-class classifier, we have developed a multi-class solution, and to address the class-imbalanced dataset, we have taken images from different datasets available online. One main challenge faced during our development is mainly to improve the stability of the DGAN model during the training phase. To analyse the performance of GAN, we have developed two CNN models in parallel based on the architecture of ResNet50 and VGG16 by augmenting the training datasets using the traditional rotation, flipping, and scaling methods. We have used both labelled and unlabelled data for testing to test the models. DGAN has outperformed the conventional data augmentation by achieving a performance of 91.1% for the unlabelled dataset and 92.3% for the labelled dataset. On the contrary, CNN models with data augmentation have achieved a performance of up to 70.8% for the unlabelled dataset. The outcome of our DGAN confirms the ability of the model to learn from unlabelled datasets and yet produce a good diagnosis result.

## 1. Introduction

According to Tizek et al. [1], one of the most common health problems affecting people of all ages worldwide is skin diseases. Acknowledging that many of these diseases can be treated nowadays, the burden of skin problems is still significant. A Bulletin of the World Health Organization in 2005 states that skin diseases have a significant impact on people's quality of life, causing lost productivity at work and school and discrimination due to disfigurement [2]. Given the rise in the prevalence, seriousness, and consequence of skin diseases worldwide, studies and research are carried out periodically to help analyse and reveal the patterns, twists, and statistics about these diseases. The global burden of skin diseases is analysed in a study carried out by Coffeng et al. [3]. This study shows that skin diseases are responsible for 1.79% of the global burden of disease, measured in disability-adjusted life years (DALYs), that is, the number of years lost due to ill-health disability early death due to 15 skin conditions in 188 countries. The findings reveal that dermatitis turned out to be responsible for the most global DALYs with a total burden of 0.38% followed by acne vulgaris (0.29%), psoriasis (0.19%), urticaria (0.19%), viral skin diseases (0.16%), fungal skin diseases (0.15%), scabies (0.07%), melanoma (0.06%), pyoderma (0.05%), cellulitis (0.04%), carcinoma (0.03%), decubitus ulcer (0.03%), and alopecia areata (0.01%).

Presently, most of the conclusions on skin problem cases are drawn mainly based on skin doctors' or dermatologists' years of experience or their subjective analysis, which is not all the time guaranteed to be free of misjudgement. A very high level of expertise is needed to differentiate between, for example, two fungal infections since they have pretty much the same symptom growth type. It is not that obvious to diagnose a skin disorder considering the number of factors to be considered, namely the skin lesion morphology, colour, type of growth, and the different symptoms. According to Onsoi et al. [4], many misdiagnose skin disorders. Furthermore, due to this enormous reliance on practitioners and their costly consultation and physical examination fees, many people tend to neglect or fail to afford medical care for their skin.

Despite the alarming statistics, skin disorders have received relatively little attention worldwide. Computer-aided software can help diagnose skin problems, and the results might be more reliable and reproducible. The recent development in image processing and deep learning in the medical field has raised interest in exploring its application in detecting skin diseases. So far, there is limited research conducted on deep learning in detecting and diagnosing skin problems. However, given the good performance of similar applications in other medical domains, there are scopes in exploring deep learning techniques to detect skin problems. In addition, the training of deep learning models, which need large datasets, provides more research direction for exploring ways of overcoming the challenges of limited labelled datasets.

## 2. Related Work

Based on human anatomy studies by Doctors of Medicine, Hoffman [5], and Stöppler [6], the skin is the largest body organ that covers the whole human body with an average surface area of about 20 square feet and an average weight of 6 pounds. However, despite being considered the first line of defence of the human body, the skin is not utterly resistant. Subsequently, the skin is constantly prone to various external and genetic factors. As a result, skin diseases affect people worldwide, irrespective of their ages, skin colour, living conditions, or socioeconomic status. However, a recent study, the Skin Cancer Index 2018, shows that geographical and geopolitical factors make skin cancer occurrences more common and sometimes deadly in particular regions over others [7].

Researchers are developing computer-aided applications to automate the process of skin problem detection [8–12]. Techniques have been devised to perform the core processes of image capturing, preprocessing, segmentation, feature extraction, and image classification. Clinical image capture can be obtained using nonstandard cameras, mobile phones, and digital cameras [13, 14]. Dermoscopy can equally be used to capture skin images. Dermoscopic images have the advantages of bright lighting conditions and a considerable low noise level [15]. To detect the skin lesion, Ünver and Ayan [16] have applied the YOLOv3 model in dermoscopic images. The ISBI 2017 dataset was utilised for training the classifier in this work. This technique produces a bounding box that can then extract the coordinates.

To enhance the quality of the images before processing, Ünver and Ayan and Hajgude et al. [16, 17] have applied the adaptive median filter. Hajgude et al. [17] have classified lesions from normal skin images using multilevel thresholding using the Otsu method. Vineela et al. [18] adopted the region-based segmentation for skin cancer detection. On the other hand, Amarathunga et al. have applied a threshold-based segmentation method to separate healthy skin from the affected skin. This work adopted morphological operations to remove objects of the same type, such as noise in the background and foreground. The watershed algorithm was applied to identify the disease area of the skin. When extracting features from skin lesion images, features such as colour, texture, and shape are generally used since these are the only properties ruling in the lesion area [19–22]. Several classification techniques such as the support vector machine (SVM), the K-nearest neighbor (k-NN), the minimum distance from mean (MDM), and the convolutional neural network (CNN) have been tested in several previous skin disease detection projects (Bhattacharya). CNN is currently spurring interest in its application in the medical domain as it has demonstrated outstanding capabilities and has achieved a satisfactory level of accuracy. Boman and Volminger [23] have distinguished melanoma from seborrheic keratosis and solar lentigo using a deep convolutional neural network to classify skin cancer. The initial results showed that the authors could classify benign and malignant melanoma. In the same line, Shanthi et al. [24] have used CNN on the DermNet database, where four types of diseases, namely acne, keratosis, eczema herprticum, and urticaria, were considered. They used only 30 to 60 samples for each class. Deep learning requires a considerable amount of data to reach a reasonable performance. Since there are limited skin disease datasets, most applications use pretrained CNN models and apply transfer learning.

Automated skin disease detection applications are complex to develop because of the different variations such as the skin tones, location of the disease, and types of image acquisition equipment. In addition, multi-class classification is challenging as skin problems have distinct characteristics. On the other hand, CNN has attained excellent results in the medical field as in other fields and thus provides hope in developing automated medical systems [30, 31]. Generative adversarial network (GAN), yet another technique, is attracting the attention of researchers since it can model complex real-world image data. It also can restore balance in imbalanced datasets [32]. However, so far, only a few applications have adopted GAN for the data augmentation along with binary classification only [33].  Table 1 analyses the existing work in this field, which eventually identifies the research gap. To contribute to developing a robust skin cancer detection and classification application, we have explored the capability of GAN on our dataset. We have developed an enhanced CNN in addition to transfer learning.  Section 3 shows the architecture of the proposed model.  Section 4 details the development of the solution while the evaluations of the work are exposed in Section 5.

The main contributions of this study are as follows:

•Construction of a custom deep learning generative adversarial network (DGAN) to overcome the challenges of limited labelled datasets. DGAN uses the CNN as generator and discriminator model, thus providing a dense network for an efficient classification.
•Training of the DGAN model and achieving a good level of stability.
•Building of two custom enhanced CNN models by fine-tuning the required parameters and applying traditional data augmentation.
•Evaluation of DGAN and traditional data augmentations.

## 3. Materials and Methods

### 3.1. Datasets

There are several datasets that are available online for research purposes. However, they vary in terms of the types of skin diseases that they capture. Since several types of skin diseases (see Figure 1) are being considered, namely acne, vulgaris, angioma, carcinoma, keratosis, nevus, café-au-lait macule, dermatofibroma, eczema, keloid, psoriasis, dermatitis ulcer, steroid acne, versicolor, heat rash, and vulgaris, a new dataset has been constructed. Images have been taken from the PH2 [34], SD-198 [35], Interactive Atlas of Dermoscopy [36], and DermNet dataset (https://apps.lib.umich.edu/database/link/11961). The *PH*^2^ dataset has 200 dermoscopic images, of which 40 are melanoma and 160 are nevus cases. On the other hand, SD-198 dataset is a clinical skin lesion dataset comprising 6584 clinical images of 198 skin diseases. Interactive Atlas of Dermoscopy contains more than 1000 clinical cases with both clinical and dermoscopic images. DermNet stores 23 types of skin diseases with a total of 19,500 images. Images in the PH2 dataset were in bitmap (BMP) format and were converted in JPEG format. However, it is to be noted that resolutions vary from image to image and from category to category. A new dataset was constructed by randomly taking images from the 4 mentioned datasets for each skin problem considered in this study. The total number of images in the dataset was 13,650.  Table 2 lists the number of images that have been considered for each type of skin disease. In this research, for each skin disease category, half of the images were labelled and the rest were unlabelled.

## 4. Development

### 4.1. Image Preprocessing

Several techniques can be used for image preprocessing to convert the image into an appropriate format for later processing and remove noise and artefacts that may be present in the image. In the first instance, image scaling, which resizes the images to a specific width pixel [37], is being applied, followed by colour space transformation. Since colour information is critical in skin disease detection systems, attempts are made to withdraw the most convenient colour of images for advanced processing, as proposed by Al-Jumailya et al.. Next, contrast adjustment techniques are applied to enhance the brightness of dark images. Since the images for the model training were chosen from different online dermatology resources and may be of various sizes and colour spaces, image scaling and colour space transformation were adopted to rescale all images to standard image size and colour space. In this phase, all the images will be converted into RGB space, the standard Internet colour system, and the default colour standard of digital cameras. After analysing the potential image restoration techniques, the median filter followed by the Gaussian filter was utilised to smooth the images. This was also useful to lower the effect of small elements such as thin hairs that are sometimes present in the skin lesion images.  Table 3 presents a list of notations to understand equations used in this article.

### 4.2. Data Augmentation Using Deep Generative Adversarial Networks (GANs)

Figure 2 shows the high-level architecture of proposed solution. Deep learning is gaining more popularity in image classification and can extract and select more features than traditional methods [38, 39]. However, large annotated datasets are required to gain from the potentials of deep learning. Unfortunately, it is observed that there are many unlabelled datasets in real life, which requires professional experts for the annotations. Recently, one appealing method that emerged is the GANs. Udrea and Mitra [40] have used GANs for training skin images and have classified them into pigmented and nonpigmented lesions. In other medical applications for diabetic retinopathy, Lim et al. [41] have generated GAN images for data augmentation. The performance had shown significant improvement compared with when GANs were not utilised. Motivated by these recent developments, GAN has been explored in our work. GANs are generative models that generate samples similar to the training dataset by learning the true data distribution. It uses deep learning methods, such as convolutional neural networks (CNNs). It classifies the test samples based on the reconstruction error instead of compressing the input into a latent space. GAN consists of two sub-models: the generator and the discriminator [42]. The generator produces fake samples. It attempts to generate the realistic samples that belong to the training sample. On the other hand, the discriminator model attempts to distinguish the true images from the generator's fake samples, thus reprimanding the generator for producing unrealistic samples [33, 41].  Figure 3 illustrates the architecture of the GANs. Mathematically, the generator's weights are optimised to maximize the probability that fake data are classified as belonging to the real data. The discriminator's weights are optimised to maximize the probability that the real input data are classified as real while minimising the probability of fake input data being classified as real. In a given *d* dimensional space, for *x* ∈ *R*^d^, *y*=*P*_data_(*x*) is a mapping from *x* to real data *y*. The two networks can be described as a min-max game with the following equation:

(1) $$\begin{array}{c} \underset{G^{\prime }}{\min}\underset{D}{\max}V\left(G,D\right)=E\left(\log\left\{1-D\left[G\left(x\right)\right]\right\}\right). \end{array}$$

The first part of (1) shows the log probability of the discriminator predicting that the input sample is genuine, and the second half reflects the probability of discriminator predicting that the generator's output is not genuine. We have trained our model until the optimal situation is reached, that is, when an output obtained from the generator (*G*) cannot be concretely labelled by the discriminator (*D*) as real or fake, showing that the networks cannot be improved further. We have built the generator and discriminator to implement our deep learning GAN (DCGAN). In this work, we have used a noise vector having 100 elements from a Gaussian distribution as input termed as *x*. We have used a noise vector with 100 elements from a Gaussian distribution as an input in this work. We have considered a limited number of images from each class representing skin diseases. Well-trained GAN should give the impression of generating real data samples from noise vectors.

### 4.3. Generator

We have constructed the generator using four up-sampling layers to double the size of the image. We have five convolution layers and have used the ReLU function for the activation layer. The architecture is illustrated in Figure 4. First, an arbitrary space is created, which is a 100-element Gaussian random number to produce an output of 2D array with 32 × 32 × 3. In the deep GAN, the first layer has enough nodes to represent a low-resolution version of the image, that is, 16 × 16 × 3 or 8 × 8 × 3. From several experiments conducted, we have considered 16 × 16 × 3. Thus, the first dense layer represents 256 × 16 × 16. The activations from these nodes are then reshaped to pass into a convolution layer, 16 × 16 × 256, having 256 different 16 × 16 feature maps. The next part is to up-sample the low-resolution image to a higher resolution version. A stride of 2 × 2 was used. This process was continued until a 32 × 32 output was obtained. The output layer has three filters, and the “same” padding was used to preserve the dimension of 32 × 32 × 3 pixels. The tanh activation was used in the last layer so that the output falls within [−1,1]. Conv_2D_3_256 represents the function up-sampling also known as deconvolution, meaning that there are 256 convolutional neurons, having a filter of 3 × 3. FC in Figure 4 denotes the fully connected layer.

### 4.4. Discriminator

The discriminator outputs the score of a sample belonging to the real dataset or the synthetic dataset. It is to be noted that the discriminator's training sample consists of both real sample from the original dataset and the fake samples that have been generated from the generator. Our discriminator consists of 5 dense layers as shown in Figure 5. The classifier has 4 convolution layers with max-pooling layers. The ReLU function was used for each layer except where sigmoid function was applied for the last layer to map the output value to the range [0, 1]. The discriminator uses max-pooling of stride 2, with a filter size of 2 × 2.

### 4.5. Training of the Model

First of all, the generator makes a prediction on a batch of noise samples. Initially, the generator initialises a set of weights and the output is eventually meaningless values, as shown in Figure 6.

While training, we want the discriminator to think that the output of the image by the generator is real. Back propagation is used to update the model's weights to allow the generator to produce good fake images. Thus, the discriminator inputs a set of samples. The first half represents the output from the generator and the second half represents samples from the real datasets, as illustrated in Figure 7. The discriminator is trained so that the discriminator can distinguish between real and fake skin problem images. Note that this process was done for each class of skin problem.

First, the weights of the discriminator are frozen. Then, we feed the generator with random noise and allow the GAN to output a probability. The value would be less than 0.5 as expected as the output of the discriminator was set close to 0 if it is not genuine. Now, we make the GAN understand that the outcome should be 1. In this case, the results in the errors are being propagated to the generator. The generator's weights are then tuned with every sample in the batch to make the output of the GAN close to 1. In this way, the generator learns to produce skin problem samples that resemble real skin problem images. This process is repeated for every batch on the training set.

### 4.6. Hyperparameter Fine-Tuning

As illustrated in Figure 5, dropout is being used [43]. This process prevents our model from overfitting. After several experiments, we have used NAdam [44] over AAdam [45] for our optimiser using default parameters, except for the learning rate. The latter was updated at each epoch as in [46]. The binary cross-entropy loss function was used with a batch size of 30.

## 5. Results and Discussions

### 5.1. Performance of DCGAN

We have trained the generator and the discriminator from scratch; while inspiring the promising results, GAN has achieved in different applications [33, 41, 47]. This implementation uses Keras API on TensorFlow for modelling. We have used Python, which is hosted on the Anaconda development platform. The images were preprocessed as described earlier, and some of the resulting images after applying the filters are illustrated in Figure 8.

Both the discriminator and the generator were trained. Then, the training loss of both the generator and discriminator was analysed and is displayed in Figure 9. The loss convergence towards the end shows that the GAN model has reached optimality. The optimised model is used to classify the images. 70% of the original datasets were considered for the training and 30% for testing each class of images. Note that 30% of images were taken as unlabelled data.  Table 4 demonstrates the accuracy of each class of images using DCGAN. The accuracy can be computed using the following equation[48]:

(2) $$\begin{array}{c} \text{accuracy}=\frac{SD+SR}{SD+SR+GD+GR}, \end{array}$$

where *SD* be the true positive, *SR* be the true negative, *GD* be the false positives, and *GR* be false negatives.

For example, of 300 images of keratosis, our model could correctly classify 265 images. Likewise, 235 of 240 steroid acnes were correctly classified. The overall accuracy of the model is 91.1%. The precision of the model has also been computed and is computed based on the (3). The precision of the overall model is 88%.

(3) $$\begin{array}{c} \text{precision}=\frac{SD}{\text{Total Number of PR edictions}}. \end{array}$$

### 5.2. Performance of Enhanced ResNet50 and VGG16 with Data Augmentation

We have also used data augmentation and the two pretrained deep learning models, namely ResNet50 and VGG16. Data augmentation is the process of transforming each image into diverse possible ways and adding all of the augmented samples to the dataset to increase its size [49]. The applied transformations include factors or parameters such as centring, zoom, flip, shift, rotation, shear, and variations in brightness and contrast, as discussed in (Alberio et al.). In addition, Grochowski and Mikołajczyk [50] addressed that image augmentation is a technique used to address issues such as insufficient images for training or uneven class balance within datasets.  Figure 10 shows the augmentation on images, and Figure 11 represents segmented images.

We have used the architecture of the ResNet50, which consist of one convolutional layer and 16 residual modules between two pooling layers [51]. It uses 3 × 3 filters for the convolution. On the other hand, the architecture of VGG16 has 19 weight layers consisting of 16 convolutional layers with 3 fully connected layers and 5 pooling layers [52]. We have developed the models based on the architectures of the two CNN models and have trained it on the same datasets used for DCGAN. However, experiments were conducted on fully labelled datasets and partially labelled datasets as well. We have fine-tuned the parameters to reduce overfitting and have varied the learning rate at different epochs. It was tested with the same dataset used for DCGAN.  Table 4 displays the results of the two enhanced ResNet50 and VGG16 models after the application of traditional data augmentation.

Figure 12 exhibits the performance of ResNet50 and VGG16 after data augmentation with fully labelled datasets. Similarly, Figure 13 gives the interpretation for partially labelled datasets. The overall performance for ResNet50 after applying data augmentation is 70.8% and that of VGG16 is 64.9%. There is a significant difference in the overall performance of the models when using labelled and unlabelled datasets with data augmentation. This confirms the fact that data traditional data augmentation has some limitations when working with unlabelled images, which eventually impact the performance rate. A summary of our achievement is illustrated in Table 5.

### 5.3. Evaluations

As discussed in [33, 53] (Guan and Loew), CNN requires a large amount of annotated data for training a model from scratch, which is not feasible in most cases. For some time now, data augmentation is being adopted to increase the number of images in datasets. As in previous work [29, 54, 55], we have also experimented with data augmentation and CNN with both labelled and partially labelled datasets. From the results obtained, we have achieved an overall performance of 70.8% for our enhanced ResNet50 after performing data augmentation, and likewise, we have reached a performance of 64.9% for the VGG16. From the findings emanated from a research conducted on the classification of melanoma skin cancer by Budhiman et al., it was concluded that a better validation performance was obtained on a dataset without data augmentation using ResNet. This is the case in our research work, where DCGAN has achieved better results compared with the traditional data augmentation. However, in a work carried out by Ayan and Unver [16, 56] to classify melanoma, the results of the ISIC augmented dataset outperform the results of the non-augmented datasets. Nevertheless, it is observed that only two classes of data were considered. Gradually, GAN has emerged and is known to address the challenges of limited unlabelled dataset [33, 40, 47, 57]. Udrea and Mitra have achieved a validation performance of 92% for melanoma and nonmelanoma skin problem. On the other hand, a result of 86.1% was reached by Rashid et al.. Most of the work conducted focuses on two-class images. Inspired by the appealing performances and ability of GAN, the latter has been investigated and applied to our dataset. We have been able to classify 15 different types of skin problems. We have compared our work with existing research whereby GAN was also used to classify skin problem as listed in Table 6.

Rashid et al. [33] have achieved a performance of 86.1% for 7 classes of skin problem, while we have achieved an accuracy rate of 91.1% for 15 types of skin diseases. The other work listed has achieved a higher performance compared with our work. However, they have considered only two classes of images, while in our case we have developed a multi-class model for 15 types of skin problem.

From the comparison made in Table 7, Budhiman et al. have classified images into normal and cancerous, that is, 2 classes. A result of 83% was obtained without data augmentation. In this case, the ISIC dataset was enough since only 2 classes of images were required. Data augmentation was not required since the number of labelled data was sufficient for the two classes of images, and it was developed using the pretrained ResNet CNN models. On the other hand, Ayan and Unver [16] have classified melanoma into benign and malignant using a custom-built CNN model and have achieved an accuracy of 81% with data augmentation. We have achieved far better results using the DCGAN, and in addition, 15 types of skin problems have been considered.

## 6. Conclusion

In this work, we have developed two CNN models based on the ResNet50 and VGG16 architecture using data augmentation on both labelled and unlabelled datasets. We usually experiment many challenges when developing CNN models for medical applications owing to the lack of labelled datasets. At the same time, GAN is being emerged, known to be a model based on a generator and discriminator model that generates synthetic images and that classifies the test samples based on the reconstruction error. Thus, we have developed a DGAN for the classification of 17 classes of skin problems. We have trained the model and fine-tuned the parameters to make the GAN stable, which is a great challenge when developing such applications. The performance achievement for our multi-class classification has reached 92.3%, showing its capabilities of working with unlabelled datasets, outperforming the results achieved when using traditional data augmentation. As a future direction, more experiments should be conducted to analyse the performance of GAN for multi-class classification and to determine the ways to make GAN stable to improve its performance. It is equally important to test with different types of data with many variations in terms of illuminations, colour, texture, among others.

## Figures and Tables

**Figure 1:** Type of skin disease. (a) Acne. (b) Nevus. (c) Angioma. (d) Eczema. (e) Dermatitis ulcer. (f) Heat rash.

**Figure 2:** High-level architecture of the proposed solution.

**Figure 3:** Architecture of GANs.

**Figure 4:** Architecture of generator.

**Figure 5:** Architecture of discriminator.

**Figure 6:** Architecture of generator.

**Figure 7:** Model training.

**Figure 8:** Examples of preprocessed images.

**Figure 9:** Training loss of generator and discriminator.

**Figure 10:** Data augmentation on images.

**Figure 11:** Application of segmentation on images.

**Figure 12:** Performance of ResNet50 and VGG16 after data augmentation with fully labelled datasets.

**Figure 13:** Performance of ResNet50 and VGG16 after data augmentation with partially labelled datasets.

**Table 1:** Comparison of the state-of-the-art methods.

Authors	Techniques	Datasets used	Performance and observation
Hameed et al. [25]	Pretrained AlexNet model	9,144 images obtained from different sources available online	Done multi-class classification for healthy, acne, eczema, benign, or malignant melanoma. A recognition rate of 86.21% was reached. The authors have catered for overfitting using k-folds
Bi et al. [26]	A probability-based stepwise integration (PSI) approach for segmentation refinement	ISBI 2016, ISBI 2017 and PH2 dataset	Able to segment melanomas with fuzzy boundaries and heterogeneous textures compared with other work conducted so far. However, the main focus is on the segmentation process
Al-Masni et al. [27]	Deep full-resolution convolutional networks	Public datasets: ISBI 2017 and *PH*^2^	Skin lesion segmentation using convolution network. An overall segmentation accuracy of 94.03% for the ISBI 2017 test dataset and 95.08%, respectively, for the PH2 dataset. However, the authors have worked until the segmentation of the lesions only
Yuan and Lo [28]	Enhanced convolutional-deconvolutional networks	ISBI 2017 skin lesion segmentation challenge, trained on 2000 images	Worked on the segmentation process only
Ünver and Ayan (2019) [16]	You Only Look Once (YOLO) and the GrabCut algorithm	*PH* ^2^ and the ISBI 2017	A recognition rate of 90% challenges in the segmentation process because of the presence of other artefacts such as hairs, bubbles, and ruler marks
Sun et al. [15]	Handcrafted techniques and VGGNet	SD-198	Used VGGNet and has achieved a performance of VGGNet of 50.27%. The authors have analysed the performance of handcrafted techniques and deep techniques. The authors have concluded that the performance is different when using labelled datasets and real unlabelled datasets
Wu et al. [11]	Pretrained EfficientNet-B4 CNN algorithm	Own created dataset consisting of 4,740 clinical images	A diagnosis assistant was built based on the pretrained model. An overall diagnostic accuracy of 95.8% was achieved. However, no work has been conducted with respect to overfitting, and there was no analysis of the hyperparameters that may influence performance when using CNN
Budhiman et al. [29]	ResNet without data augmentation	ISIC 2018	Used the architecture of ResNet50, ResNet40, ResNet25, ResNet10, and ResNet7 models for training the datasets. Experiments were conducted with and without data augmentation. The validation accuracy achieved was 83% on data without data augmentation

**Table 2:** Number of images for each skin disease.

Type of skin disease	Number of images
Acne vulgaris	900 (450 labelled and 450 unlabelled)
Angioma	1200 (600 labelled and 600 unlabelled)
Carcinoma	800 (400 labelled and 400 unlabelled)
Keratosis	1000 (500 labelled and 500 unlabelled)
Nevus	1100 (550 labelled and 550 unlabelled)
Café-au-lait macule	900 (450 labelled and 450 unlabelled)
Dermatofibroma	950 (475 labelled and 475 unlabelled)
Eczema	1200 (600 labelled and 600 unlabelled)
Keloid	800 (400 labelled and 400 unlabelled)
Psoriasis	900 (450 labelled and 450 unlabelled)
Dermatitis ulcer	750 (375 labelled and 375 unlabelled)
Steroid acne	800 (400 labelled and 400 unlabelled)
Versicolor	750 (375 labelled and 375 unlabelled)
Heat rash	800 (400 labelled and 400 unlabelled)
Vulgaris	900 (450 labelled and 450 unlabelled)

**Table 3:** List of notations.

Notation	Description
*x*	Gaussian distribution as input and is
*R* ^*d*^	Real data in a given *d* dimensional space
*y*	Output
*P*_data_	Mapping function from *x* to real data *y*
*G*	Generator function
*D*	Discriminator function
*V*	Value function of the generator and discriminator together to a minimax game
*SD*	True positive
*SR*	True negative
*GD*	False positives
*GR*	False negatives

**Table 4:** Performance of model using DCGAN.

Class of skin disease	Number of test images	Accuracy (%)
Acne vulgaris	270	92.1
Angioma	360	89.2
Carcinoma	240	92.1
Keratosis	300	88.7
Nevus	330	96.6
Café-au-lait macule	270	91.3
Dermatofibroma	285	83.2
Eczema	360	86.4
Keloid	240	94.2
Psoriasis	270	96.0
Dermatitis ulcer	225	82.4
Steroid acne	240	98.3
Versicolor	225	93.5
Heat rash	240	82.5
Vulgaris	270	90.2

**Table 5:** Summary of overall performance.

GAN		Data augmentation			
Performance (%) (labelled dataset)	Performance (%) (unlabelled dataset)	Performance (%) (labelled dataset)		Performance (%) (unlabelled dataset)	
		ResNet50	VGG16	ResNet50	VGG16
92.3	91.1	85.9	80.2	70.8	64.9

**Table 6:** Comparison of state-of-the-art techniques.

Authors	Number of classes	Technique	Accuracy (%)
Rashid et al. [33]	7 types of skin lesions	GAN	86.1
Ali et al. [57]	2 classes (malignant and benign melanoma)	DCGAN	91.9
Sedigh et al. [53]	2 classes (malignant and benign melanoma)	GAN	71.1
Udrea and Mitra [40]	2 classes (pigmented vs. nonpigmented lesions)	DCGAN	92.1
Proposed work	15 types of skin diseases	DCGAN	91.1

**Table 7:** Existing work using CNN models.

Authors	Details	Technique	Accuracy (%)
Budhiman et al. [29]	ResNet50 on ISIC 2018	ResNet50 without data augmentation	83
Ayan and Unver [16]	CNN on ISIC 2018	CNN with data augmentation	81

## Data Availability

The ISBI 2017 and PH2 datasets data used to support the findings of this study are included within the article.
